# A Protocol for the Diagnosis of Autism Spectrum Disorder Structured in Machine Learning and Verbal Decision Analysis

**DOI:** 10.1155/2021/1628959

**Published:** 2021-03-30

**Authors:** Evandro Andrade, Samuel Portela, Plácido Rogério Pinheiro, Luciano Comin Nunes, Marum Simão Filho, Wagner Silva Costa, Mirian Caliope Dantas Pinheiro

**Affiliations:** University of Fortaleza (UNIFOR)-Graduate Program in Applied Informatics, Av. Washington Soares, 1321-Bl J Sl 30-60.811-905 Fortaleza, Brazil

## Abstract

Autism Spectrum Disorder is a mental disorder that afflicts millions of people worldwide. It is estimated that one in 160 children has traces of autism, with five times the higher prevalence in boys. The protocols for detecting symptoms are diverse. However, the following are among the most used: the Diagnostic and Statistical Manual of Mental Disorders, 5th Edition (DSM-5), of the American Psychiatric Association; the Revised Autistic Diagnostic Observation Schedule (ADOS-R); the Autistic Diagnostic Interview (ADI); and the International Classification of Diseases, 10th edition (ICD-10), published by the World Health Organization (WHO) and adopted in Brazil by the Unified Health System (SUS). The application of machine learning models helps make the diagnostic process of Autism Spectrum Disorder more precise, reducing, in many cases, the number of criteria necessary for evaluation, denoting a form of attribute engineering (feature engineering) efficiency. This work proposes a hybrid approach based on machine learning algorithms' composition to discover knowledge and concepts associated with the multicriteria method of decision support based on Verbal Decision Analysis to refine the results. Therefore, the study has the general objective of evaluating how the mentioned hybrid methodology proposal can make the protocol derived from ICD-10 more efficient, providing agility to diagnosing Autism Spectrum Disorder by observing a minor symptom. The study database covers thousands of cases of people who, once diagnosed, obtained government assistance in Brazil.

## 1. Introduction

In a society where competitiveness is a substantial differential in profile and productive capacity, any severe psychological disorder that an individual may present constitutes a factor of their exclusion from the wealth-generating process. In this context, individuals with Autism Spectrum Disorder (ASD), as well as other severe psychological disorders, are observed with reticence from an early age and, often, discriminated against in daycare centers, schools, universities, and companies where they try to get an insert. A probable cause for this discrimination is based on the lack of information about ASD and other psychological disorders, as well as on the lack of conscience of the potential contribution that every human being can give to society, especially when there is an appreciation of the plurality of ideas and points of view.

According to the World Health Organization (WHO), ASD is a mental disorder that affects more than 70 million people worldwide. Worldwide estimates show one child with autism every 160 [1], with a prevalence five times higher among boys. In Brazil, there is a ratio of one autistic child for every 360. Although considered underestimated, Brazil's data show that there is a significant demand for specialized care [2]. Currently, the need for effectiveness and efficiency in diagnosing ASD goes beyond just health since people diagnosed with this disorder also seek to participate in selective processes for the formation of work teams. These diagnoses can help these people in both the educational and professional placement in the job market. On the other hand, the globalized world requires competitiveness and sustainability from companies, which depend heavily on people. In their selection processes, companies seek to select healthy professionals and, often, have excluded those who suffer from specific problems, such as ASD, even though they have different skills.

As a social contribution, the present study is aimed at applying a machine learning model to make the ASD diagnostic process more precise and concise, reducing the number of criteria necessary for the evaluation. To this end, the study proposes a hybrid approach, based on the juxtaposition of machine learning algorithms, aimed at knowledge discovery, associated with a multicriteria method of decision support based on Verbal Decision Analysis (VDA). The general objective is to evaluate how the hybrid methodology now proposed can make the protocol derived from the International Classification of Diseases, 10th edition (ICD-10) more efficient, enabling the diagnosis of Autism Spectrum Disorder by observing a minor symptom. The study sought to link the ICD-10 with the codes and structure of the DSM-5, aiming at expanding the understanding and diagnosis capacity from different clinical points of view. This objective comes considering that the hybrid model proposal mentioned above is applied to ASD and considering that mental disorders are the main focus of the Diagnostic and Statistical Manual of Mental Disorders, 5th Edition (DSM-5).

Moreover, to validate the hybrid model, the study used a database provided by the Social Security Technology and Information Company of Brazil-DATAPREV. Mentioned data refer to thousands of cases of people who obtained the assistance benefit related to ASD, as provided by Brazil's federal legislation. The granting of these benefits goes through evaluating each case of children with ASD, to whom the Benefit of Continuous Provision (BPC) program applies. These assessments have an extensive questionnaire divided into Social Assessment and Medical-Expert Assessment, which allowed for research to obtain more consistent data on the stages of medical and social evaluation.

This article is divided into five sections. After the introduction, the study presents the second section that outlines the systematization of the fundamental theoretical basis on which the work is based. The third section describes the methodology used, which is subdivided into four subsections—which deal, respectively, with the database, the Random Forest machine learning algorithm, the applied learning framework, and the Verbal Decision Analysis (VDA) method addressed. The fourth section presents the results achieved. Finally, the fifth section concludes the work and proposes actions and perspectives for future work.

## 2. Theoretical Reference

This section contains some important topics about Autism Spectrum Disorder and highlights proposed information technology solutions used to support the diagnosis and referral of that disorder.

### 2.1. Highlights about Autism Spectrum Disorder Concepts

Autism Spectrum Disorder (ASD) consists of a neurodevelopmental disorder characterized by patterns of stereotyped and repetitive behaviors and difficulty in communication and social interaction. There are several protocols for diagnosing the disease. The most widely adopted are the Diagnostic and Statistical Manual of Mental Disorders, 5th Edition, known as DSM-5, from the American Psychiatric Association; the Revised Autistic Diagnostic Observation Schedule (ADOS-R); the Autistic Diagnostic Interview (ADI); and the International Classification of Diseases and Health-Related Problems (ICD-10), a criterion published by the World Health Organization (WHO) and adopted in Brazil by the Unified Health System (SUS). In Figure 1, there is a highlight of the Autism Spectrum Disorder (ASD) in the context of the Neurodevelopmental Disorders categorization, as discriminates in the DSM-5.

Scientific investigations about Autism Spectrum Disorder have evolved a lot since the beginning of the last century, in both the theoretical and empirical aspects. From this perspective, it is clear that since the term “autism” was coined by the psychiatrist Eugen Bleuler, in 1911, when analyzing symptoms of schizophrenic patients, including the disclosure of other autistic patterns by Hans Asperger, in 1970, research has advanced considerably. With the passage of time and the deepening of knowledge on the subject, the expression Autism Spectrum Disorder (ASD) started to feature a very different set of behavioral changes with early onset, chronic course, and variable impact in multiple areas of development [4].

Furthermore, Martone and Santos-Carvalho [5] performed a bibliographic review of the articles published by the *Journal of Applied Behavior Analysis* (JABA) between the years 2008 and 2012, focusing on the importance of verbal behavior for the detection of the disorder [5]. Cohen et al. [6] present a pioneering study in which it uses a neural network to classify the disorder. The results showed the importance of implementing new technologies in the detection of the disorder and, simultaneously, pointed to the need to better explore the application of neural networks, with all its variations of parameters, to improve the classification of ASD [6].

### 2.2. Information Technology Solutions Used in the Diagnosis of Autism Spectrum Disorder

Following the technological approach, Yekta et al. [7] proposed an ASD diagnostic system, called the Autism Screening Expert System (ASES), whose main attributes or criteria were chosen from the use of machine learning techniques on a basis obtained by questionnaires. In this case, to select the diagnosis's main attributes, the technology solution “Random Forests and Support Vector Machines” was used. This system seems to be very efficient for detecting the disorder in children aged 2 to 6 years [7]. In a similar approach, Khullar et al. [8] developed a system—the Handheld Expert System (HES)—to diagnose ASD using artificial neural networks. It obtained 100% (one hundred percent) accuracy in detecting the disorder when considering the protocol described in the Diagnostic and Statistical Manual of Mental Disorders (DSM-5) [8]. Also, in this same line, Nunes et al. [3] present an intelligent solution based on a hybrid model of the expert system associated with the multicriteria method MACBETH (Measuring Attractiveness by a Categorical Based Evaluation Technique) to support the early diagnosis of ASD in children aged up to two years [3].

In a similar context, Cohen [9] presents a study of a neural network that simulates and shares formal qualitative similarities with selective attention and the generalization of deficits observed in people with autism. In simulations in which the model was taught to discriminate children with autism from children with mental retardation, there were observations that neuropathologies described in the literature are sufficient to explain some of the unique pattern recognition and learning skills, as well as their generalization and acquisition problems [9]. Florio et al. [10] show the importance of a second opinion on the diagnosis of ASD and the use of technology to provide independent clinical evaluation, increasing diagnosis accuracy. Challenges related to using technology to offer independent second opinions include the possibility for individuals and relatives to participate in self-diagnosis activities [10].

Still, from the perspective of intelligent systems, Thabtah [11] points out that ASD has been studied in the area of the behavioral sciences using intelligent methods based on machine learning to speed up the screening time or improve the sensitivity, specificity, or precision of the diagnostic process. In this sense, machine learning considers the problem of ASD diagnosis as a classification task, by which predictive models are built based on historical cases and controls. These models must be connected to a screening tool to achieve one or more of the objectives. This work sought to shed light on recent studies that use machine learning in the ASD classification to discuss its pros and cons. It highlighted a noticeable problem associated with current ASD screening tools: the reliability of these tools using the DSM-IV rather than the DSM-5 manual. As a result, the need to change the current screening tools to reflect the newly imposed criteria for ASD classification in the DSM-5 has been suggested, particularly the diagnostic algorithms incorporated in these methods [11].

In the same sense, Thabtah [12] states that machine learning is a multidisciplinary research topic that employs intelligent techniques to discover relevant hidden patterns used in forecasting to improve decision-making. Thus, some machine learning techniques, such as Random Forests and others, were applied to datasets related to autism to build predictive models. These models claim to increase clinicians' ability to provide robust ASD diagnostics and prognosis [12].

In a systematic review, Thabtah and Peebles [13] evaluated and critically analyzed 37 different ASD screening tools to identify possible areas that need to be addressed through further development and innovation [13].

In another analysis, Thabtah et al. [14] proposed a new machine learning framework related to screening autism for adults and teenagers containing vital characteristics. The results obtained reveal that the machine learning technology was able to generate classification systems with acceptable performance in terms of sensitivity, specificity, and precision, among others [14].

On the other hand, in a different approach, Neto et al. [15] presented the G-ASD, which consists of a prototype of a game to assist professionals in the field of psychology using the methodology of Applied Behavior Analysis (ABA) in teaching children's learning with Autism Spectrum Disorder (ASD) [15]. The G-ASD shows how important the use of games is in the process of building the knowledge of children with autism, assisting the professional in teaching colors to autistic children. From a social and pedagogical perspective, Lampreia [16] evaluates the official instruments for the diagnosis of autism and comments that, due to the intention of unifying them, it harms some areas such as social interaction, communication, interests, and development activities. Costa et al. [17] address the difficulty of including autistic people in the information technology segment and highlight information for analysis and discussion regarding the inclusion of autistic people in higher education and the respective job market in the area of information technology.

Several approaches are promoted to study neurological disorders. Maenner et al. [18] investigated the Random Forest algorithm in a set of autism data from the Georgia Autism and Developmental Disabilities Monitoring (ADDM) network, using phrases and words obtained in child development assessments. The dataset consists of 5,396 assessments for 1,162 children, of which 601 are on the spectrum. Random Forest classifiers were assessed on an independent test dataset that contained 9,811 evaluations from 1,450 children. The results reported that the Random Forest reached about 89% of the predictive value [18].

Finally, it is observed that the Random Forest algorithm has been used with an outstanding frequency in decision-making processes in the health area, mainly for ASD diagnosis and treatment. This was one of the main reasons for using the Random Forest in the present study as an algorithm that is part of the hybrid model now proposed.

## 3. A Methodology for the Autism Spectrum Disorder Diagnostic Protocol

The present study used the quantitative research method, looking for numbers, frequency of characteristics, and quantifiers in the responses to social and medical assessments of children diagnosed with ASD, candidates for the Benefit of Continuous Provision (BPC) of Social Security in Brazil. Also, a qualitative approach was used to interpret the results of the evaluations in the Brazilian medical-social context.

The study database was obtained from the Social Security Technology and Information Company of Brazil-DATAPREV. The said database has 320,302 (three hundred twenty thousand three hundred two) records referring to the responses in the medical evaluations of 3,861 (three thousand eight hundred sixty-one) children from 0 to 5 years old, from all over Brazil, representing 82 (eighty-two) social, environmental, and clinical variables. This base is fed from evaluation forms, whose items can be transformed into labels for the variables that characterize diseases. By mapping the main characteristics, it is possible to assign a response to each question. The variables include information about the person's identity, the socioenvironmental aspects, and the clinical criteria necessary to identify ASD. The process of preparing the model proposal can be summarized in the following steps:

- In the first stage, after collecting the responses in the evaluations, the characteristics were organized with keywords (tag) and related to the respective qualifiers in a data table (Analytical Base Table (ABT))
- Then, in the second stage, the data were classified using the machine learning algorithm, Random Forest, which combined several decision trees to obtain a prediction with greater accuracy and stability
- The third stage consisted of the creation of a form with the nine most used characteristics for the application by the decision-makers
- Finally, in the fourth stage, the ZAPROS-IIIi method, implemented in the ARANAÚ tool [19], performed the Verbal Decision Analysis (VDA), aiming at the order of preference of the main characteristics of the ASD

These characteristics constitute the proposed model.

Figure 2 presents a summary of the process of the steps described above, providing a simplified view of the creation of the proposed hybrid model mentioned.

### 3.1. Preparation for Processing

There are two preprocessing steps. The first one was developed to appropriate the data for manipulation in the Orange framework, which uses the machine learning model (see step I and step II, in Figure 2). The second one was developed, from the first preliminary result, to adjust the information for the Verbal Decision Analysis (see step III, in Figure 2).

In the first preprocessing stage, the questionnaire, received in a .txt extension, has the questions classified and labeled. After transposition, they are arranged in tabular form, in a panel format. The answers are mapped and assigned to the item, with a specific weight, ranging from 0 to 4. The resulting file has the extension .csv and is consumed by the machine learning framework.

In the second preprocessing step, the result of the model imported will be the shortest path in the decision tree, in which nodes have represented the symptoms of the disorder investigated. Such a way will again be converted into a questionnaire, with each sign being a variable that is the subject of a question, with 3 (three) evaluation criteria, each with 3 (three) possible qualitative answers. The result will serve as input to the Verbal Decision Analysis method, ZAPROS-IIIi, implemented in the ARANAÚ tool [19].

### 3.2. Random Forest Method Considerations

Random Forests are randomized decision trees capable of predicting expected values of regressions and classifications. The model was published by Breiman [20, 21], and since then, the technique has become an important data analysis tool, quite versatile and with few adjustment parameters. In this sense, despite its simplicity, the method is generally recognized for its precision and ability to handle small sample sizes, large resource spaces, and complex data structures [22]. The versatility of the algorithm contributed to the popularity of Random Forests, in addition to having few parameters to adjust. Many practical issues have successfully involved Random Forests, including forecasting air quality, chemoinformatics, ecology, 3D object recognition, and bioinformatics, to name a few. Many have validly proposed variations of the original algorithm to improve calculation times while maintaining good forecasting accuracy. Breiman's Random Forests were also extended to quantile estimation, survival analysis, and ranking forecast [22].

Regarding the theoretical aspect, the analyses are less conclusive, and, regardless of their extensive use in practical contexts, little is known about the mathematical properties of Random Forests. To date, most studies have focused on isolated parts or simplified versions of the procedure. The most famous theoretical result is that of Breiman [20, 21], which offers an upper limit to the error of generalization of forests in terms of correlation and strength of individual trees. It was followed by a technical note [22], which focuses on a modified version of the original algorithm. A critical step was subsequently followed by Jeon and Lin [23], who established lower limits for nonadaptive forests, independent of the training set [22]. They also highlighted an interesting connection between Random Forests and a specific class of predictors of *k*-nearest neighbors (KNN) that was further developed [22].

The nature of the procedure can explain the difficulty in adequately analyzing Random Forests, the former being a subtle combination of different components. Among the essential ingredients of the forest, both bagging (Breiman [24, 25]) and classification and regression trees (CART) criterion (Breiman et al. [26, 27]) play a critical role. Bagging, like a bootstrap-aggregating contraction, is a general aggregation scheme that proceeds by generating subsamples of the original dataset, building a predictor for each resampling, and deciding on the mean. It is one of the most useful computationally intensive procedures to improve unstable estimates, especially for large data and high-dimensional datasets, where it is impossible to find a suitable model in one step due to the complexity and scale of the problem [22]. The most influential CART algorithm by Breiman et al. [26, 27] originated the CART-split selection, used in the construction of individual trees to choose the best cuts perpendicular to the axes. In each node of each tree, the best cut is selected, optimizing the CART division criterion, based on the notion of Gini impurity (classification) and quadratic regression error [22].

However, despite the essentiality of the algorithm components mentioned above, both bagging and CART are challenging to analyze, which is why theoretical studies have considered simplified versions of the original procedure. This analysis is usually done by simply skipping the bagging step and replacing the CART partition selection with a more elementary cutting protocol. Also, in Breiman's Random Forests, each leaf—that is, a terminal node—of the individual trees contains a preestablished fixed number of observations (this parameter is usually chosen between 1 and 5). Thus, the authors opt for simplified and independent data procedures, thus creating a gap between theory and practice [22].

Motivated by the discussion, Scornet et al. [22] studied some asymptotic properties of Breiman's algorithm [20, 21] in additive regression models. These researchers proved the consistency of Random Forests, which provides a first basic theoretical guarantee of efficiency for this algorithm. This finding was the first consistency result for Breiman's [20, 21] original procedure. The approach was based on a detailed analysis of the cell's behavior generated by the selection of the CART-split as the sample size increased. The study also showed that Random Forests could adapt to a sparse structure when the dimension is large, but only a smaller number of coordinates make the information.  Figure 3 describes the Random Forest algorithm [22].

The general structure consists of the regression in which a random input vector *X* ∈ [0, 1]^*p*^ is observed, where “*p*” is the dimension of the vector. The objective is to predict the integrable random response square *Y* ∈ *R* by estimating the function of regression *m*(*x*) = *E*[*Y* | *X* = *x*]. Therefore, it is assumed that the training sample is given by *D*_*n*_ = (*X*_1_, *Y*_1_), ⋯, (*X*_*n*_, *Y*_*n*_) in  [0, 1]^*p*^ × *R*, independently distributed as the independent pair (*X*, *Y*). The objective is to use the dataset *D*_*n*_ to construct an estimate *m*_*n*_ : [0, 1]^*p*^ → *R* of the function “*m*.” Thus, it is said that an estimated regression function *m*_*n*_ is consistent if *E*[*m*_*n*_(*X*) − *m*(*X*)]^2^ → ∞, where the expectation *E* is greater than *X* and *D*_*n*_ [22].

A Random Forest is a predictor that consists of a collection of *M* trees of random regression. For the *j*-th family tree, the predicted value at query point *x* is indicated by *m*_*n*_(*x*, Θ_*j*_, *D*_*n*_), where Θ_1_, ⋯, Θ_*M*_ are independent random variables, distributed as a generic random variable *Φ* and independent of *D*_*n*_. In practice, this variable is used to resample the training set before the growth of individual trees and to select successive directions for separation. The trees are combined to form the finite estimate of the forest [22].

(1) $$\begin{array}{c} m_{M,n}\left(x,\Theta_{1},\cdots ,\Theta_{M},D_{n}\right)=\frac{1}{M}\overset{M}{\underset{j=1}{\sum }}m_{n}\left(x,\Theta_{j},D_{n}\right). \end{array}$$

Since one can choose, in practice, *M* as large as possible, Scornet et al. [22] demonstrated the property; according to which, the infinite forest estimate obtained as the limit of equation (1) is verified as follows when the number of *M* trees grows to infinity [22]:

(2) $$\begin{array}{c} m_{n}\left(x;D_{n}\right)=E_{\Theta }\left[m_{n}\left(x,\Theta ,D_{n}\right)\right], \end{array}$$

where *E*_Θ_ denotes the expectation in relation to the random parameter Θ, conditional on *D*_*n*_. The law of large numbers, which states that it almost certainly depends on *D*_*n*_, justifies this operation [22]:

(3) $$\begin{array}{c} \underset{M\to \infty }{\lim}m_{n,M}\left(x;\Theta_{1},\cdots ,\Theta_{M},D_{n}\right)=m_{n}\left(x;D_{n}\right). \end{array}$$

See Breiman [20, 21] for more details. From now on, to simplify the notation, *m*_*n*_(*x*) will be written instead of *m*_*n*_(*x*; *D*_*n*_) [22].

In the original forests of Breiman [20, 21], each node of a single tree is associated with a hyperrectangular cell. At each stage of the tree's construction, the set of cells forms a partition [0, 1]^*p*^. The root of the tree is [0, 1]^*p*^ itself, and each tree grows, as explained in Algorithm 1 in Figure 3. This algorithm has three parameters [22]:

1. *m*_try_ ∈ {1, ⋯, *p*}, which is the number of preselected directions for the tree's dividing
2. *a*_*n*_ ∈ {1, ⋯, *n*}, which is the number of data points sampled in each tree
3. *t*_*n*_ ∈ {1, ⋯, *a*_*n*_}, which is the number of leaves in each tree

By default, in the original procedure, the parameter *m*_tinytry_ is set to *p*/3, *a*! is set to *n* (resampling is done with substitution), and *t*_*n*_ = *a*_*n*_. However, in this approach, resampling is done without replacement, and the parameters *a*_*n*_ and *t*_*n*_ may differ from their default values [22].

The algorithm works by growing *M* different trees as follows. For each tree, data points are drawn at random without replacing the original dataset; then, in each cell of each tree, a division is chosen maximizing the CART criterion; finally, the construction of each tree is interrupted when the total number of cells in the tree reaches the value *t*_*n*_. Therefore, each cell contains exactly one point in the case *t*_*n*_ = *a*_*n*_ [22].

### 3.3. Framework Orange Canvas

Demsar et al. [28] designed a framework called Orange, used in the present work. The framework is a set of machine learning and data mining tools for data analysis through Python scripts and visual programming. Orange is intended for experienced users and programmers, as well as data mining students. It is based on the C++ language; however, it allows developers to work with the Python language.

### 3.4. Considerations about the ZAPROS-IIIi Verbal Decision Analysis Method

Verbal Decision Analysis (VDA) assumes that most decision-making problems can be expressed in natural language and consists of the decision-making process based on the related representation of the problem [29]. It is also noteworthy that this methodology addresses unstructured problems, characterized by the absence of logical and well-defined procedures to be applied to its resolution [29]. These problems are qualitative and are complex to be organized, formalized, and measured numerically. Also, it is not possible to have all the information necessary to resolve them. Thus, the analysis process is also subjective, which requires the collection of information from the decision-maker.

According to Larichev and Moshkovich [29], the methods that make up the structure of Verbal Decision Analysis are ZAPROS-III, ZAPROS-LM, PACOM, and ORCLASS, as well as their characteristics and applications. The analysis of a large amount of data by humans has shown that the correct way of operating is used by the mentioned methods and works as follows [29]:

1. Comparison of two assessments on a verbal scale by two criteria
2. Assignment of multicriteria alternatives to decision classes
3. Comparative verbal evaluation of alternatives according to separate criteria

The mentioned methods are Decision Support Systems (DSS) that help a decision-maker to classify alternatives of multiple attributes. The Verbal Decision Analysis framework's first three methods are aimed at establishing a ranking of the alternatives in order of preference. The latter presented is the only methodology for classification based on the VDA structure.  Figure 4 shows an easy visualization of several Verbal Decision Analysis methodologies according to the types of problems.

For this work, the ZAPROS-IIIi method will be applied. The method fits the characteristics of the problem addressed, which allows the structuring of a decision rule used to compare the alternatives and will not be changed, even if the set of alternatives is modified and applies to problems with a large number of alternatives. The ZAPROS-III method is structured in three well-defined main stages: formulation of problems, elicitation of preferences, and comparison of alternatives. As proposed in the main version of the ZAPROS method, the method is aimed at classifying alternative criteria in scenarios that involve minimal set criteria and criteria values and a large number of alternatives. The relevant criteria and their values for decision-making and the scale of preferences based on the preference of the decision-maker are obtained in the first and second stages. In the last step, the comparison between the alternatives based on the decision-maker's preferences is performed. These stages are described below.

As part of the Verbal Decision Analysis structure as well, the ZAPROS-III methodology can be considered an evolution of ZAPROS-LM. Similar to the ZAPROS-LM and PACOM methods, this method is aimed at classifying a group of alternatives, from the most preferable to the least preferable.

Although ZAPROS-III applies a similar procedure to obtain the preferences of its successor, it implements modifications that make it more efficient and more accurate concerning inconsistencies. The number of incomparable alternatives is substantially less than in the previous ZAPROS.

Figure 5 presents a flowchart with the steps to apply the VDA ZAPROS-IIIi method. According to the scheme described in the procedure, it is possible to divide the application of the method into three stages: formulation of the problem, elicitation of preferences/validation of the decision-maker's preferences, and comparison of alternatives.

Since there is an exponential growth in the alternatives of the problem and the growth of the necessary information in the process of obtaining preferences, a disadvantage of the method is that to control the complexity, the number of criteria and values of the treated criteria is limited. The ZAPROS-IIIi methodology brings an essential difference in relation to the previous models: the division into different stages. The method proposes that the two substations are transformed into one instead of basing the decision-maker's preferences on the first reference situation and then establishing another preference scale using the second reference situation. Therefore, the questions asked considering the first reference situation are the same as those asked considering the second reference situation. Thus, both situations will be considered in answering the question at the same time. The change implies process optimization: dependence on criteria is avoided.

Ultimately, these modifications increased method comparability so that several alternatives defined as incomparable, when applying the ZAPROS method purely, could now be compared directly or indirectly. Furthermore, these changes in the method process did not change its computational complexity [30].

Considering that it is complicated for a decision-maker, the process of ordering preferences, Tamanini et al. conducted a study with data from a battery of tests for patients with a possible diagnosis of Alzheimer's disease to structure a decision tree based on the characteristics that led to the determination of that disease. In this study, the preference scale was established through the analysis of the resulting tree and, subsequently, the scale was subjected to the ZAPROS method to classify the tests involved in the case studied [31]. This hybrid model shows the potential of integrating VIDA with machine learning solutions [32].

## 4. A Protocol to Determine the Main Characteristics for Diagnosing Autism Spectrum Disorder

The model was structured using decision trees with the Random Forest to classify the main characteristics of medical evaluations. Then, these characteristics were submitted to the VDA ZAPROS-IIIi method to be placed in order of preference of the decision-maker. The construction of the protocol, structured in machine learning and the ZAPROS-IIIi method of VDA, used the criteria defined based on each qualifier of obstacles experienced by individuals with ASD, namely [33]:

*Mild/moderate (from 0% to 49% commitment)*. Has a slight, regular barrier or difficulty.

*Severe (from 50% to 95% commitment)*. Has high or extreme difficulty.

*Complete (96% to 100% commitment)*. Has a barrier or total difficulty.

The evaluations of 3,861 (three thousand eight hundred sixty-one) children aged 0 to 5 years were selected, indicating the classification “F84” and family of the ICD-10, which characterizes the global developmental disorders—this classification in the ICD-10 corresponds to the code “299.00” in the DSM-5. After data collection, it had the use of keywords for each of the characteristics of the social and medical evaluations, aiming at generating the ABT (Analytical Base Table) and executing the Random Forest, using Orange.  Figure 6 shows the configuration for using the Random Forest.

### 4.1. Identification of the Main Characteristics of the Diagnosis of Autism Spectrum Disorder

The evaluation of the sample of 3,861 (three thousand eight hundred sixty-one) cases, using the decision tree, made it possible to identify the following characteristics [33, 34]:

- Functions of speech fluency and rhythm (changes in fluency, stuttering, verbiage, dyslalia-tachylalia, and bradylalia, among others), in a way compatible with the age group-b330
- Difficulty to intentionally use the sense of sight (follow objects visually, observe people, watch a sporting event, and observe people or children playing, among others), in a manner compatible with the age group-d110 from 1 year
- Difficulty in acquiring and executing necessary skills (using cutlery and pencils, among others) and complex skills (games, sports, using tools, and watching, among others), in a way compatible with the age group-d155 from 2 years
- Sleep functions (start, maintenance, quantity, and quality of sleep), in a way compatible with the age group-b134
- Memory functions (recent, remote, and amnesic memory disorders), in a way compatible with the age group-b144 from 3 years old
- Global psychosocial functions (interpersonal skills necessary for the establishment of reciprocal social interactions, in terms of meaning and purpose, adaptability, responsiveness, predictability, persistence, and accessibility, and interpersonal interactions, among others), in a manner compatible with the age group-b122 from 2 years
- Difficulty moving using specific equipment or device to facilitate movement (walker, wheelchair, crutches, cane, and others), in a manner compatible with the age group-d465 from 3 years old
- Difficulty walking (moving on foot, for short or long distances, without the aid of people, equipment, or devices), in a manner compatible with the age group-d450 from 2 years
- Vision functionalities (quality, acuity, light and color perception, monocular and binocular vision, myopia, hyperopia, astigmatism, hemianopsia, presbyopia, color blindness, tunnel vision, central and peripheral scotoma, diplopia, night blindness, and adaptability to light, among others), in a way compatible with the age group-b210

Figure 7 shows the resulting tree of the Orange application, with five levels, and the alternatives considered in the assessment. These main characteristics were applied to the ZAPROS-IIIi method, implemented in the ARANAÚ tool, for an ordering of the most preferable to the least preferred characteristic, in the answers for cases of ASD diagnosis.

Based on the characteristics identified early in Section 4.1, a form was prepared to be filled out by decision-makers in a survey format.  Table 1 presents these characteristics in the form of a questionnaire. Each question in this questionnaire had answers under three criteria discriminated in the lines of Table 1, namely:

*A*. Voice, mental, or vision functions must present a barrier or difficulty.

*B*. Learning and the application of knowledge must present a barrier or difficulty.

*C.* Mobility must present a barrier or difficulty.

In the sequence, each of these criteria was evaluated under the following three alternatives discriminated and identified in the columns of Table 1:

*Complete (96% to 100% commitment)*. Has a barrier or total difficulty.

*Severe (from 50% to 95% commitment)*. Has high or extreme difficulty.

*Mild/moderate (from 0% to 49% commitment)*. Has a slight, regular barrier or difficulty.

The mentioned questionnaire served as a basis for conducting research with a sample of 91 (ninety-one) professionals with knowledge and experience in the treatment of people who have ASD:

- 74 (seventy-four) health professionals, twenty doctors, forty physiotherapists, forty nurses, four psychologists, four speech therapists, and two occupational therapists
- 17 (seventeen) professionals in the educational field

After the elicitation phase, each professional's preferences in the research generated the results shown in Table 1, which were compared with the results obtained through decision trees. Then, the data with values of criteria and alternatives, acquired in the research, were loaded in the ARANAÚ tool to define the order of preference of the main characteristics and their qualifiers most likely to determine the definitive diagnosis for ASD. The table in Figure 8 shows the order of preference of the ASD's main characteristics, established by the ZAPROS-IIIi method, implemented in the ARANAÚ tool after processing the data obtained in the research. These data enabled the combination of vectors formed by “criteria × alternatives,” that is, “rows × columns” of Table 1. The graphical representation in Figure 8 makes it possible to observe that the characteristics most preferable to decision-makers have more outgoing arcs than incoming arcs.

## 5. Conclusion and Future Work

The present study made it possible to analyze the questions of social and medical assessments of the Benefit of Continuous Provision (BPC) applied to children with Autism Spectrum Disorder.

The evaluations have an extensive questionnaire. With the application of decision support methods, it was possible to simplify the choice of specific characteristics for faster and more accurate diagnosis, taking into account the importance of early diagnosis since most of the cases are still detected later. With that, there was a speed gain in identifying the disease, facilitating the physician's decision-making.

This work presented a structured protocol, using decision trees with the Random Forest to classify the main characteristics of the evaluations and the ZAPROS-IIIi method for ordering these characteristics.

The first phase of the study demonstrated that the main symptoms—considered variables or vertices of the tree graph constructed by the Random Forest—are the following, in summary: speech dysfunction, difficulty in intentionally using vision, trouble in acquiring and executing basic and complex skills, sleep dysfunction, memory dysfunction, global social dysfunctions, difficulty moving, difficulty walking, and difficulty in vision. Also, the next step, based on Verbal Decision Analysis, resulted in the following ordering of the criteria selected in the previous step, namely:

- 8. For the difficulty in walking (moving on foot, for short or long distances, without the aid of people, equipment, or devices), in a way compatible with the age group-d450 from 2 years old
- 6. For global psychosocial functions (interpersonal skills necessary for the establishment of reciprocal social interactions, in terms of meaning and purpose, adaptability, responsiveness, predictability, persistence, and accessibility, and interpersonal communications, among others), in a manner compatible with the age group-b122 from 2 years
- 7. For the difficulty of moving using specific equipment or device to facilitate movement (walker, wheelchair, crutches, cane, and others), in a manner compatible with the age group-d465 from 3 years
- 1. Regarding the functions of fluency and rhythm of speech (changes in fluency, stuttering, verbiage, dyslalia-tachylalia, and bradylalia, among others), for a definite diagnosis of ASD-b330
- 4. For sleep functions (start, maintenance, quantity, and quality of sleep), in a way compatible with the age group-b134
- 9. For vision functions (quality, accuracy, light and color perception, monocular and binocular vision, myopia, hyperopia, astigmatism, hemianopsia, presbyopia, color blindness, tunnel vision, central and peripheral scotoma, diplopia, night blindness, and adaptability to light, among others), in a way compatible with the age group-b210 and age group-d465 from 3 years old
- 2. For the difficulty of intentionally using the sense of sight (following an object visually, observing people, and watching a sporting event or children playing, among others), for a definite diagnosis of ASD-d110
- 3. For the difficulty in acquiring and executing necessary skills (using cutlery and pencils, among others) and complicated skills (games, sports, using tools, and watching, among others), in a way compatible with the age group-d155 from 2 years old
- 5. For memory functions (recent, remote, and amnestic memory disorders), in a way compatible with the age group-b144 from 3 years old

The overall result suggests that of the more than 80 (eighty) variables evaluated, only 9 (nine) would be sufficient to indicate the diagnosis of Autism Spectrum Disorder safely.

The authors suggest, for future work, the application of a broader approach to the protocol, conducting future research in the universe of children and adolescents from 0 to 18 years old, and a more in-depth analysis of the characteristics and their qualifiers.

A comparative study of the present protocol proposal with another model, using algorithms based on Bayesian networks, logistic regression, or other machine learning techniques, will expand and improve the model now proposed for the decision-making process. At this point in the study, comparisons can be made between the mentioned algorithms [34].

## Figures and Tables

**Figure 1:** Neurodevelopmental Disorders, according to DSM-5. Source: Nunes et al. [3].

**Figure 2:** The graph with the processing structure of the proposed hybrid model. Source: formatted by the author.

**Figure 3:** The Random Forest algorithm. Source: Scornet et al. [22].

**Figure 4:** Verbal Decision Analysis methodologies. Source: Nunes et al. [3].

**Figure 5:** Procedure for applying the ZAPROS-IIIi method. Source: Pinheiro et al. [30].

**Figure 6:** Configuration for using Random Forest. Source: formatted by the author.

**Figure 7:** The sampling of the main alternatives considered in the evaluation of the resulting tree. Source: formatted by the author.

**Figure 8:** Order of preference among the main characteristics of ASD. Source: formatted by the author.

**Table 1:** The main characteristics of ASD.

According to your experience and assessment for early diagnosis of Autism Spectrum Disorder (ASD) in children up to 5 years of age, evaluate the following:				
Questions	Criteria	Alternatives		
		1. Complete	2. Severe	3. Mild/moderate
1. Regarding the functions of fluency and rhythm of speech (changes in fluency, stuttering, verbiage, dyslalia-tachylalia, and bradylalia, among others), for a definite diagnosis of ASD-b330, you believe that:	A	6	54	31
	B	5	42	44
	C	6	32	53
2. For the difficulty of intentionally using the sense of sight (following an object visually, observing people, and watching a sporting event or children playing, among others), for a definite diagnosis of ASD-d110, you believe that:	A	9	44	38
	B	1	43	47
	C	4	36	51
3. For the difficulty in acquiring and executing necessary skills (using cutlery and pencils, among others) and complicated skills (games, sports, using tools, and watching, among others), in a way compatible with the age group-d155 from 2 years old, do you believe that:	A	5	43	43
	B	4	42	45
	C	10	28	53
4. For sleep functions (start, maintenance, quantity, and quality of sleep), in a way compatible with the age group-b134, do you believe that:	A	7	42	42
	B	10	39	42
	C	6	49	36
5. For memory functions (recent, remote, and amnestic memory disorders), in a way compatible with the age group-b144 from 3 years old, you believe that:	A	12	43	36
	B	7	39	45
	C	7	30	54
6. For global psychosocial functions (interpersonal skills necessary for the establishment of reciprocal social interactions, in terms of meaning and purpose, adaptability, responsiveness, predictability, persistence, and accessibility, and interpersonal communications, among others), in a manner compatible with the age group-b122 and age group-b125 from 2 years, do you believe that:	A	22	41	28
	B	19	46	26
	C	8	36	47
7. For the difficulty of moving using specific equipment or device to facilitate movement (walker, wheelchair, crutches, cane, and others), in a manner compatible with the age group-d465 from 3 years, you believe that:	A	6	50	35
	B	5	54	32
	C	4	39	48
8. For the difficulty in walking (moving on foot, for short or long distances, without the aid of people, equipment, or devices), in a way compatible with the age group-d450 from 2 years old and age group-d465 from 3 years, you think that:	A	10	41	40
	B	6	47	38
	C	23	40	28
9. For vision functions (quality, accuracy, light and color perception, monocular and binocular vision, myopia, hyperopia, astigmatism, hemianopsia, presbyopia, color blindness, tunnel vision, central and peripheral scotoma, diplopia, night blindness, and adaptability to light, among others), in a way compatible with the age group-b210 and age group-d465 from 3 years old, you think that:	A	7	35	49
	B	2	44	45
	C	13	49	29

Source: formatted by the author.

## Data Availability

The data used to support the findings of this study are available from the corresponding author upon request.
